The article "A Cohort Study of the Effects of Integrated Medical and Nursing Rounds Combined with AIDET Communication Mode on Recovery and Quality of Life in Patients Undergoing Percutaneous Coronary Intervention" was published in 2022. Journal: Comput Math Methods Med.

# A Cohort Study of the Effects of Integrated Medical and Nursing Rounds Combined with AIDET Communication Mode on Recovery and Quality of Life in Patients Undergoing Percutaneous Coronary Intervention

**DOI:** 10.1155/2022/9489203

**Published:** 2022-08-24

**Authors:** Lan Li, Yongheng Li, Tao Yin, Jinglin Chen, Fengjiao Shi

**Affiliations:** ^1^Department of Cardiovascular Medicine II, The Fourth Hospital of Changsha City, No. 70 Lushan South Road, Yuelu District, Changsha City, Hunan Province, China 410006; ^2^Nursing Department, The Fourth Hospital of Changsha City, No. 70 Lushan South Road, Yuelu District, Changsha City, Hunan Province, China 410006; ^3^Respiratory Medicine Ward II, The Fourth Hospital of Changsha City, No. 70 Lushan South Road, Yuelu District, Changsha City, Hunan Province, China 410006

## Abstract

**Objective:**

To explore the influence of the communication mode of “Acknowledge, Introduce, Duration, Explanation, and Thanks (AIDET)” on the postoperative recovery and quality of life of patients undergoing percutaneous coronary intervention.

**Methods:**

Sixty patients with percutaneous coronary intervention in our hospital from April 2019 to April 2021 were selected. The patients were randomly divided into a control group (*n* = 30) and research group (*n* = 30). The control group received integrated medical and nursing rounds, and the research group received integrated medical and nursing rounds combined with AIDET communication mode. The scores of nursing satisfaction, cardiac function, self-nursing ability, short-term prognosis, and quality of life were compared between the two groups.

**Results:**

In the comparison of nursing satisfaction between the two groups, the satisfaction of the research group was low in 1 case, moderate in 6 cases, and high in 27 cases, with a satisfaction rate of 96.67%. In the control group, there were 7 cases with low satisfaction, 10 cases with moderate satisfaction, and 13 cases with high satisfaction, with a satisfaction rate of 76.67%. The nursing satisfaction of the research group was higher than that of the control group, and the difference was statistically significant, and the difference was statistically significant (*P* < 0.05). After intervention, the cardiac function of the two groups was improved. The LVEF and LVESVI of the research group were higher than those of the control group, while the WMSI of the research group was lower than that of the control group (*P* < 0.05). In the comparison of self-nursing ability, the self-nursing maintenance, self-nursing management, self-nursing confidence, and total score of self-nursing in the research group were significantly higher than those in the control group, and the difference was statistically significant (*P* < 0.05). The incidence rates of acute myocardial infarction (AMI), revascularization, arrhythmia, heart failure, cardiogenic shock, and cardiac death in the research group were obviously lower than those in the control group, and the difference was statistically significant (*P* < 0.05). After intervention, the scores of quality of life of the two groups decreased, and the scores of physiological function, psychological function, social function, and health self-cognition in the research group were lower than those in the control group (*P* < 0.05).

**Conclusion:**

Medical and nursing integrated ward rounds combined with AIDET communication mode can effectively improve the prognosis of patients undergoing percutaneous coronary intervention to promote the establishment of a harmonious nurse-patient relationship. The patients' self-care ability is able to be effectively enhanced.

## 1. Introduction

With the development of economy, society, and medical technology, the disease-centered traditional medical model has been gradually replaced by the “bio-psycho-social” medical model. “Bio-psycho-social” is a person-centred medical model. At this time, there is an urgent need for hospital management to use the spirit of innovation to explore a new working mode to adapt to the gradual transformation of the health care relationship from the initial dominant-subordinate model to the juxtaposition-complementary model [1]. In the past, the working mode was that doctors instructed nurses to work and nurses carried out medication orders. Therefore, there was a lack of comprehensive communication between doctors and nurses. In the 1950s, the nursing activities of senior practical nurses were carried out in Britain, the United States, and other developed countries. The work mode of combining medical and nursing assistance has been applied in clinical work, which can well improve the quality and efficiency of medical and nursing service to meet the expectations of each other's roles between doctors and nurses. The integration model of medical and nursing assistance has sprung up and has been gradually promoted [2]. The mode of integration of medical care and assistance is different from the previous way in which doctors make medical plans and nurses carry out doctor's orders, which breaks the original parallel lines of doctors and patients and nurses and patients [3]. In 2003, the American Nursing Association defined the health care integration model as a reliable cooperation model between doctors and nurses [4]. At the same time, there is a reasonable division of labor, close contact, information exchange, and mutual cooperation between doctors and nurses [5]. It is an important part of the continuous improvement of medical quality. The studies have shown that good cooperation between doctors and nurses can shorten the days of hospitalization, reduce the incidence of mortality and complications, and improve nursing satisfaction [6–8].

The quality of communication not only affects patients' medical experience but also can be used as one of the important reference indicators to evaluate and judge the quality of medical services [9]. The use of certain tools or skills will help to improve the efficiency of communication and solve clinical practical medical and nursing problems. Since the 1990s, foreign scholars have begun to study the mode of doctor-patient communication. Studer Group was founded in 1999, which provided guidance, teaching, evidence-based tools, and strategies to health care organizations and rural hospitals in the United States to help medical organizations achieve cultural transformation [10]. In AIDET communication mode, A (acknowledge) is indicated as greetings. I (introduce) is indicated as introduction, in which your name, professional title, qualification, and working hours are introduced. D (duration) is indicated as process. In view of the following operational matters and how much time it will take, the patients have an expectation of the operation to ease their anxiety about unknown things and to better cooperate with our work. E (explanation) means letting patients know that our services represent their interests. T (thanks) means thank you. At the end of the operation, the patients will be grateful for their cooperation and understanding, which not only shows the good professionalism of the medical staff but also allows the patients to get rid of their helplessness as a patient and restore their sense of self-worth. Finally, they are informed that if they need help, they can contact us at any time. The use of AIDET communication mode helps to communicate clearly and improve the patient experience [11, 12].

Percutaneous coronary intervention (PCI) refers to the treatment of cardiac catheterization to dredge the narrow or even occluded coronary artery lumen so as to improve myocardial perfusion. Although the clinical application of PCI has been mature, there is still a risk of postoperative complications, affecting the outcome of postoperative disease. Good nursing measures can play the effect of adjuvant therapy. At present, the nursing interventions of patients after PCI at home and abroad mainly include community nursing, collaborative nursing, home nursing, continuous nursing, and so on. China has also carried out some research in this area, but there are still some shortcomings [13]. Most of them only carry out health education for diseases, the form of intervention is single, and targeted guidance is lacking. The participants are only nurses; with lack of medical cooperation and good communication, patients passively receive health education given by medical staff. Medical staff do not know the relevant knowledge of patients after PCI. The duration of good self-care behavior established in life is limited [14]. At present, medical and nursing integration mode and AIDET communication mode have been used in peritoneal dialysis, wound treatment, outpatient examination, chronic disease management, and other fields and have achieved good results [15]. In this study, the impact of integrated medical and nursing rounds combined with AIDET communication mode was explored on the recovery and quality of life of patients after percutaneous coronary intervention.

## 2. Materials and Methods

### 2.1. General Information

Sixty patients with percutaneous coronary intervention in our hospital from April 2019 to April 2021 were selected. The patients were randomly divided into two groups: the control group (*n* = 30) and research group (*n* = 30). The control group received routine nursing, and the research group received medical and nursing care combined with AIDET communication mode. The age of control cases ranged from 43 to 80 years with an average of 63.35 ± 3.42 years, including 18 males and 12 females. The course of coronary heart disease ranged from 5 to 8 years with an average of 6.15 ± 1.44 years. The age of study cases was 44-76 years with an average of 63.55 ± 3.91 years, including 17 males and 13 females. The course of coronary heart disease ranged from 4 years to 8 years with an average of 6.11 ± 1.48 years. There was no statistical significance in the general data of the two groups. This study was approved by the Medical Ethics Association of our hospital, and all patients signed informed consent.

Inclusion criteria: (1) in accordance with the diagnostic criteria of coronary heart disease established by the interventional cardiology group of the Cardiology Branch of Chinese Medical Association [16], those who underwent PCI; (2) those who were more than 18 years old and less than 80 years old; (3) those who could understand and answer the questionnaire; and (4) those who have informed consent and voluntary participation in this study were included in the study.

Exclusion criteria: (1) those with mental illness, (2) those with other serious diseases, and (3) those who were accompanied by professional or temporary caregivers were excluded from the study.

Elimination standard: (1) those who died for any reason; (2) those who stopped participating in the research for various reasons; (3) those who failed to complete the questionnaire due to the loss of follow-up for various reasons; and (4) those who were hospitalized again during the intervention period were eliminated.

### 2.2. Methods

The control group accepted the traditional medical work mode. The patients received integrated medical and nursing rounds. The specific process of the integrated medical and nursing rounds mode is as follows. (1) During the morning meeting, all medical staff would turn over at the nurses' station to report the condition of patients in the ward. (2) Ward rounds were jointly attended by attending physicians, bed-in-charge residents, responsible nurses, therapists, and patients. The nurses reported the changes of their condition, the completion of treatment and the problems that need to be solved, and the bed-attendant supplement and put forward the next diagnosis and treatment plan. Finally, the attending physician put forward measures to solve the problems encountered and cooperated with nurses and therapists to evaluate the current diagnosis, treatment, nursing, and rehabilitation plan. The corresponding improvement methods were put forward. The nursing effect was observed after 3 months.

The research group carried out nursing intervention based on AIDET communication mode based on integrated medical and nursing assistance. The specific process of integrated medical and nursing rounds was the same as that of the control group. The AIDET communication mode was applied on this basis: (1) before the intervention, the relevant nurses formed an AIDET communication group to train the group staff on relevant knowledge, mainly for PCI-related knowledge and specific implementation measures of AIDET. (2) Implement AIDET and carry out nursing intervention around 5 main aspects of AIDET communication mode. A (greeting): take the initiative to greet patients, use honorific titles, take a positive attitude, learn about patients' knowledge about the disease and their physical condition, ask if they are not feeling well and need help, and always maintain a patient and understanding attitude. I (introduction): introduce yourself to patients, such as “Hello, I am your responsible nurse, my professional title is …. My working life is....” This paper introduces the development history of hospital cardiology and the level of specialist team, so as to eliminate strangeness and enhance trust. (3) Introduce the nursing measures in many aspects, such as postoperative diet, rehabilitation exercise, disease and medicine, and the importance of taking medicine on time and according to the doctor's advice, and emphasize the importance of postoperative nursing in promoting prognosis. D (process): let patients understand the postoperative nursing process and the problems that may be encountered in the postoperative rehabilitation process, the treatment methods currently used, and the examination, rehabilitation training, and drug taking methods that need to be carried out in the recovery phase, so as to enhance treatment confidence. E (explanation): patiently answer patients' questions, such as “Why should they take drugs for a long time” and “Why should they carry out postoperative rehabilitation training, such as respiratory function exercise,” so as to alleviate their doubts and fears and enhance their sense of trust. T (thanks): thank the patients for their support after the nursing work is completed, and ask the patients if they have any other needs. The nursing effect was observed after 3 months.

### 2.3. Observation Index

#### 2.3.1. Satisfaction

Evaluation of patient satisfaction: (1) evaluation tool: a patient satisfaction questionnaire was used. This questionnaire was a satisfaction questionnaire of discharged patients designed by Zhang Huizhi referring to the North American Hospital Consumer Evaluation Health Service and Service System (HCAHPS). The Cronbach's *α* coefficient of the internal consistency of the questionnaire was 0.84, the CVI of each item was 0.8-1.0, and the average CVI of all items was 0.98 [17]. (2) Assessment content: this questionnaire was divided into 5 dimensions with a total of 12 items, all of which are closed-ended questions, including 3 items for service attitude (questions 1, 2, and 5) and 1 item for business level (question 12), 2 items of caring for patients (items 3 and 4), 1 item of nursing management (item 6), and 5 items of health education (items 7, 8, 9, 10, and 11). (3) Evaluation method: the survey of patient satisfaction was conducted by the members of the research group trained in the AIDET communication mode course to distribute the questionnaire on the spot and take it back. (4) Evaluation standard: the Likert 5-level scoring method was used, which was expressed according to the degree of satisfaction, from “very satisfied” to “very dissatisfied” and from very satisfied to very dissatisfied. Five to 1 point was assigned, respectively. The score range was 12-60: ≤35 as low satisfaction, 36-53 as medium satisfaction, and ≥54 as high satisfaction. Satisfaction rate = (medium satisfaction + high satisfaction)/total number.

#### 2.3.2. Cardiac Function Index

The indexes of cardiac function, including left ventricular ejection fraction (LVEF), left ventricular end-systolic volume index (LVESVI), and wall motion integral index (WMSI), were evaluated before and 3 months after nursing.

#### 2.3.3. Self-Care Behavior

The self-nursing behavior ability was evaluated before nursing and 3 months after nursing. The SCHFI scale was developed from the University of Pennsylvania Reigel in 2004 by the self-management scale [18]. The scale had 22 items, including 3 subscales as self-nursing maintenance (10 items), self-nursing management (6 items), and self-nursing confidence (6 items). Each subscale can be used separately. Except for the two items of self-nursing management using the Likert 5-point score (0—unaware, 1—slow, 2—faster, 3—fast, and 4—very fast), the rest were rated using the Likert 4-point score (1—never, 2—occasionally, 3—often, and 4—always or daily). The standard score of each subscale can be calculated according to the formula. And the conversion formula of the standard score was as follows: standard score = (actual score − the lowest score of the item)/(the highest score of the item − the lowest score of the item) × 100. The score of each scale can be converted into 100 points. The total score of the scale was 300 points. More than 70 points in each scale indicated that the patient has better self-care ability.

#### 2.3.4. Short-Term Prognosis

Major adverse cardiovascular events (MACE) were recorded as poor prognosis, including recurrent acute myocardial infarction (AMI), revascularization, arrhythmia, heart failure, cardiogenic shock, and cardiogenic death.

#### 2.3.5. Quality of Life Scale

The quality of life scale consisted of four subscales, including physical, psychological, social, and health self-awareness with a total of 29 items [19]. Cronbach's *α* coefficient of the scale is 0.79 to 0.91. The scale was scored by 1-5 grades.

### 2.4. Statistical Analysis

SPSS23.0 statistical software was adopted to process the data. The measurement data were presented as $\bar{x}\pm s$. The group design *t*-test was adopted for the comparison, and the analysis of variance was adopted for the comparison between multiple groups. The Dunnet *t*-test was adopted for comparison with the control group. The counting data were presented in the number of cases and the percentage, the *χ*^2^ test was adopted for comparison between groups, and the bilateral test was employed for all statistical tests.

## 3. Results

### 3.1. Comparison of Nursing Satisfaction

In the comparison of nursing satisfaction between the two groups, the satisfaction of the research group was low in 1 case, moderate in 6 cases, and high in 27 cases, with a satisfaction rate of 96.67%. In the control group, there were 7 cases with low satisfaction, 10 cases with moderate satisfaction, and 13 cases with high satisfaction, with a satisfaction rate of 76.67%. The nursing satisfaction of the research group was largely higher than that of the control group, and the difference was statistically significant (*P* < 0.05). All results are shown in Figure 1.

### 3.2. Comparison of Cardiac Function

After the intervention, the cardiac function of the two groups was improved. Comparison between the two groups showed that the LVEF and LVESVI in the research group were obviously higher than those in the control group. The WMSI was remarkably lower than that in the control group, and the difference was statistically significant (*P* < 0.05). All results are shown in Table 1.

### 3.3. Comparison of Self-Nursing Ability

Compared with the self-nursing ability, the self-nursing maintenance, the self-nursing management, the self-nursing confidence, and the total score of self-nursing in the research group were significantly higher than those in the control group, and the difference was statistically significant (*P* < 0.05). All results are shown in Table 2.

### 3.4. Comparison of Short-Term Prognosis

In the comparison of recent prognosis, the incidences of AMI, revascularization, arrhythmia, heart failure, cardiogenic shock, and cardiac death in the research group were considerably lower than those in the control group, and the difference was statistically significant (*P* < 0.05). All results are shown in Figure 2. The meaning of the data in Figure 2 is the quantity. The indicators in the figure are commonly used indicators to observe the short-term prognosis of the two groups.

### 3.5. Comparison of Quality of Life Scores

After intervention, the scores of quality of life of the two groups decreased, and the scores of physiological function, psychological function, social function, and health self-cognition in the research group were markedly lower than those in the control group, and the difference was statistically significant (*P* < 0.05). All results are shown in Table 3.

## 4. Discussion

Coronary atherosclerotic heart disease is a kind of heart disease caused by myocardial ischemia, hypoxia, or necrosis caused by coronary atherosclerosis, which is called coronary heart disease. According to the World Health Organization, cardiovascular disease is the leading cause of death from noncommunicable diseases [20, 21]. The number of acute myocardial infarction in China in 2016 is about 4 million, and it is estimated that the number of acute myocardial infarction in 2030 will reach about 6.1 million [22]. PCI is one of the most effective methods for the treatment of coronary heart disease, including intracoronary stent implantation, percutaneous transluminal coronary angioplasty (PTCA), and rotational grinding of atherosclerotic plaques [23]. PCI can quickly dredge the blocked coronary artery, reduce the risk of myocardial infarction, and improve the prognosis of patients. More than 500,000 patients are treated with PCI each year in the United States. Early studies have shown that the total number of cases of interventional therapy in China exceeded 660,000 in 2016. Patients with acute ST segment elevation myocardial infarction received direct PCI in more than 50,000 cases as high as 38.9% [24]. With the continuous development and maturity of PCI, the mortality rate of coronary heart disease has been continuously reduced. Previous studies have shown that PCI in the treatment of coronary heart disease can reduce surgical trauma, improve the success rate of surgery, shorten the length of hospital stay, accelerate disease recovery, and alleviate the advantages of clinical symptoms, and restoration of myocardial blood supply can effectively improve the physiological indicators of patients, thereby improving the quality of life of patients [25, 26].

PCI has the advantages of less trauma, rapid recovery, and good prognosis and can quickly dredge the occlusive or narrow lumen under special circumstances. However, PCI is also an invasive operation, and the negative emotions such as tension, fear, anxiety, and postoperative complications will affect the therapeutic effect and prognosis of patients. Therefore, strengthening the postoperative nursing care of patients undergoing PCI is the key to save the patients' lives and improve the prognosis. With the change of the medical model, communication is becoming more and more important in nursing. A public survey has shown that higher professional skills account for only 25% of the success factors in the process of communicating with patients, while good communication skills account for 75% [27–29]. Therefore, our nursing services emphasize not only professional skills but also high emotion and high EQ. At present, there are more in-depth studies on improving the communication mode and promoting the healthy development of nurse-patient relationship at home and abroad, in which AIDET communication mode is first developed by the Studer Group team and widely used by American medical institutions. It is often used to communicate between nurses and patients, helping them to achieve good results in the adjustment of patient satisfaction [30]. The model includes procedures and standard terms for communication between nurses and patients. This model consists of the initials of five very important keywords that make up the communication framework. Through this standardized communication procedure to choose the correct language to communicate effectively with patients, it is helpful to reduce the psychological pressure of patients and their stress reaction to achieve a relaxed and pleasant state.

In the United States, the communication mode of AIDET was first used in Baptist Memorial hospitals in the late 1990s. Through the survey, it was found that patient satisfaction increased from 40% to 90% [31]. AIDET communication mode was first applied to anesthetic pain management in China. In 2010, Bor et al. applied AIDET communication mode to orthopedic pain management, which not only made the pain well controlled but also enhanced the mutual trust between nurses and patients and the enthusiasm of doctors and patients to participate in pain management [32]. In 2012, the pain management team first applied the AIDET communication model to the management of postoperative analgesia [33]. The patients have high compliance and satisfaction with postoperative analgesia services. In 2014, Ji et al. reported that the application of AIDET communication model to patients undergoing gastrointestinal surgery not only improved patient compliance and satisfaction in a short period of time but also improved the efficiency of communication between nurses and patients and maximized the efficiency of communication [34]. Through AIDET communication mode, a harmonious a5nd trusting nurse-patient relationship can be gradually established [35]. AIDET communication mode is also successfully used in maternal care (giving psychological support to parturients). Through the combination of preoperative education and postoperative rehabilitation, maternal anxiety can be alleviated [36]. After a large number of related literature review, there are no reports about the application of AIDET communication follow-up model to patients after PCI [37].

In recent years, doctors and nurses have gradually changed into a working relationship of mutual assistance and cooperation. Effective cooperation between doctors and nurses can shorten the average length of stay of patients, reduce hospitalization costs, and improve hospitalization satisfaction [38]. The integrated medical and nursing model was applied to the discharge follow-up of patients with type 2 diabetes [39]. The specific method is for doctors to establish electronic files and electronic reminders for patients. Nurses carry out health education and consultation to patients. These studies show that the integrated model of health care can improve the quality of health care without increasing economic investment. Klancik et al. pointed out that the new type of health care integration refers to a kind of interpersonal relationship in which doctors and nurses communicate and cooperate with each other in 2005 [40]. The “prehospital-in-hospital-posthospital” integrated and innovative ward of Massachusetts General Hospital is established on the basis of “relationship-based care” (RBC). Attending doctors, rehabilitation doctors, nursing specialists, head nurses, and responsible nurses participate in daily rounds to discuss patients' condition and treatment, formulate nursing and rehabilitation priorities, and extend services after discharge. It can emphasize the relationship between nurses and patients, family members, doctors, and other medical staff. This model has become a nursing work mode recognized and recommended by the American Medical Association [41]. The research on the integration of health care in China started relatively late. In 1992, Zhang et al. applied the concept of “integration of health care” to nursing teaching [42]. The integrated teaching of health care can embody the holistic view of health care, which focuses on the organic connection between treatment and nursing, avoids the disconnection and repetition of the content, and strengthens students' understanding of the integrity of health care. Since then, the concept of health care integration has been introduced into clinical work to describe health care cooperation. At present, many hospitals have begun to explore a new integrated cooperation model of health care, which is mainly used in nursing personnel training, specialist disease nursing, nursing quality management, home nursing service, and so on. The implementation of the health care integration model is mainly realized through the establishment of a health care integration team, optimization of work flow, and joint health education between doctors and nurses. According to the actual situation, the weak links of the work flow are reformed and perfected and continuously optimized, so as to effectively avoid medical and nursing risks in treatment and nursing work to improve the satisfaction of patients and the degree of cooperation between doctors and nurses. With in-depth discussion of the details of high-quality nursing services, nurses become more consultants, decision-makers, and leaders. Medical and nursing cooperation strengthens the communication among doctors to improve the work efficiency of both doctors and nurses [43]. Doctors, nurses, and patients can all benefit from the integrated work mode of health care. Therefore, the implementation of medical and nursing integration model in general hospitals is an effective means to realize the sustainable development strategy of nursing management.

Related studies pointed out that self-care ability is the premise and basis of carrying out the above-mentioned activities, such as self-examination of symptoms and signs, taking medicine according to doctor's advice, healthy diet, and proper exercise after PCI [44]. The implementation of AIDER communication mode nursing in multiple departments can improve patients' experience, relieve anxiety, and harmonize nurse-patient relationship. The reason is that most PCI patients have a long course of disease before operation and suffer from pain for a long time. Some patients are accompanied by other basic diseases, which have a great impact on the daily activities of patients, resulting in poor self-care awareness and self-care ability. At the same time, the disease will lead to self-doubt and affect the prognosis of patients. In this study, integrated medical and nursing rounds combined with AIDET communication mode were used to intervene patients after PCI in order to strengthen health education on disease-related knowledge, which make patients master postoperative nursing-related knowledge and skills. The AIDET model will pay more attention to nurses' communication attitude and skills. Through AIDET mode communication, an effective process of inertia operation is formed. The implementation of nursing measures is optimized. Integrated medical and nursing rounds combined with AIDET communication mode are effective in the intervention of patients after PCI. The reason is that integrated medical and nursing rounds can effectively avoid problems such as inconsistent medical records and disjointed medical and nursing services. Doctors and nurses should strengthen communication between the two sides and jointly understand the changes of patients' conditions and problems existing in the process of treatment and nursing. In addition, in the process of integrated medical and nursing rounds, patients' participation is also conducive to deepening their understanding of their own condition and mastering basic nursing knowledge and skills, so as to reduce the incidence of complications. Our study still has some shortcomings. Firstly, the quality of this study is limited due to the small sample size we included in the study. Secondly, this research is a single-center study, and our findings are subject to some degree of bias. Therefore, our results may differ from those of large-scale multicenter studies from other academic institutes. Our research is still clinically significant, and further in-depth investigations will be carried out in the future.

In conclusion, medical and nursing integrated ward rounds combined with AIDET communication mode can effectively improve the prognosis of patients undergoing percutaneous coronary intervention to promote the establishment of a harmonious nurse-patient relationship. The patients' self-care ability is able to effectively enhance and further improve cardiac function.

## Figures and Tables

**Figure 1:** Comparison of nursing satisfaction between the two groups.

**Figure 2:** Comparison of short-term prognosis between the two groups.

**Table 1:** Comparison of cardiac function between the two groups ($\bar{x}\pm s$).

Grouping	*N*	LVEF (%)		LVESVI (ml·m^−3^)		WMSI	
		Before intervention	After intervention	Before intervention	After intervention	Before intervention	After intervention
Control group	30	51.92 ± 3.84	55.49 ± 5.66^∗^	44.91 ± 5.32	47.14 ± 4.31^∗^	1.85 ± 0.44	1.68 ± 0.34^∗^
Research group	30	51.35 ± 3.31	59.39 ± 4.34^∗^	44.95 ± 5.44	49.19 ± 3.42^∗^	1.81 ± 0.42	1.52 ± 0.11^∗^
*t* value		0.615	2.994	0.028	2.040	0.360	2.452
*P* value		>0.05	<0.05	>0.05	<0.05	>0.05	<0.05

Note: ∗ represents the comparison before and after nursing in this group (*P* < 0.05).

**Table 2:** Comparison of self-care ability between the two groups ($\bar{x}\pm s$, points).

Grouping	*N*	Self-care maintenance	Self-nursing management	Self-care confidence	Total score
Control group	30	43.29 ± 9.32	50.39 ± 6.56	39.19 ± 4.34	135.96 ± 5.92
Research group	30	48.49 ± 5.34	58.39 ± 4.66	44.96 ± 4.10	148.65 ± 6.34
*t* value		2.651	5.445	5.293	8.012
*P* value		<0.05	<0.05	<0.05	<0.05

**Table 3:** Comparison of quality of life scores between the two groups ($\bar{x}\pm s$, points).

Grouping	*N*	Physiological function		Psychological function		Social function		Healthy self-cognition	
		Before nursing	After nursing	Before nursing	After nursing	Before nursing	After nursing	Before nursing	After nursing
Control group	30	15.75 ± 4.42	13.20 ± 2.54^∗^	16.54 ± 3.11	14.36 ± 4.66^∗^	18.84 ± 3.98	16.64 ± 2.44^∗^	15.56 ± 3.82	13.64 ± 1.55^∗^
Research group	30	15.44 ± 4.66	11.84 ± 2.31^∗^	16.45 ± 3.53	11.94 ± 1.45^∗^	18.44 ± 3.53	12.74 ± 3.42^∗^	15.75 ± 3.64	10.67 ± 2.42^∗^
*t* value		0.264	2.169	0.104	2.715	0.411	5.084	0.197	5.660
*P* value		>0.05	<0.05	>0.05	<0.05	>0.05	<0.05	>0.05	<0.05

Note: ∗ represents the comparison before and after nursing in this group (*P* < 0.05).

## Data Availability

The datasets used and analyzed during the current study are available from the corresponding author upon reasonable request.
